# Levels of Inflammatory Cytokines in Type 2 Diabetes Patients with Different Urinary Albumin Excretion Rates and Their Correlation with Clinical Variables

**DOI:** 10.1155/2013/138969

**Published:** 2013-11-14

**Authors:** Fen-qin Chen, Jiao Wang, Xiao-bo Liu, Xiao-yu Ma, Xiu-bin Zhang, Ting Huang, Dong-wei Ma, Qiu-yue Wang

**Affiliations:** ^1^Department of Geriatrics, The First Affiliated Hospital, China Medical University, Shenyang 110001, China; ^2^Department of Endocrinology, Fengtian Hospital of Shenyang Medical College, Shenyang 110000, China; ^3^Department of Endocrinology, The Fourth People's Hospital of Shenyang, Shenyang 110031, China; ^4^Department of Endocrinology, The First Affiliated Hospital, China Medical University, Shenyang 110001, China

## Abstract

Although the pathogenetic mechanism of DN has not been elucidated, an inflammatory mechanism has been suggested as a potential contributor. This study was designed to explore the relationship between low-grade inflammation and renal microangiopathy in T2DM. A total of 261 diabetic subjects were divided into three groups according to UAE: a normal albuminuria group, a microalbuminuria group, and a macroalbuminuria group. A control group was also chosen. Levels of hs-CRP, TNF-*α*, uMCP-1, SAA, SCr, BUN, serum lipid, blood pressure, and HbA1c were measured in all subjects. Compared with the normal controls, levels of hs-CRP, TNF-*α*, uMCP-1, and SAA in T2DM patients were significantly higher. They were also elevated in the normal albuminuria group, *P* < 0.05. Compared with the normal albuminuria group, levels of these inflammatory cytokines were significantly higher in the microalbuminuria and macroalbuminuria group, *P* < 0.01. The macroalbuminuria group also showed higher levels than the microalbuminuria group, *P* < 0.01. Also they were positively correlated with UAE, SBP, DBP, LDL-C, and TC. We noted no significance correlated with course, TG, or HDL-C. Only TNF-*α*; was positively correlated with HbA1c. This study revealed the importance of these inflammatory cytokines in DN pathogenesis. Further studies are needed to fully establish the potential of these cytokines as additional biomarkers for the development of DN.

## 1. Introduction 

Diabetic nephropathy (DN) has been widely recognized as a major complication associated with type 2 diabetes and is a leading cause of end-stage renal disease. It is characterized functionally by proteinuria and albuminuria and pathologically by glomerular hypertrophy, mesangial expansion, and tubulointerstitial fibrosis [1]. In recent years, our knowledge of the pathophysiological processes that lead to DN has notably improved on a genetic and molecular level. Thus, the classic view of metabolic and hemodynamic alterations as the main causes of renal injury in diabetes has been transformed significantly, with clear evidence indicating that these traditional factors are only a partial view of a much more complex picture. One of the most important changes is related to the participation of immune-mediated inflammatory processes in the pathophysiology of diabetes mellitus and its complications [2, 3]. Whether inflammation plays a role in the pathogenesis of DN and understanding what the underlying mechanisms constitute, these are questions which have yet to be answered [4, 5]. Therefore, it is very important to find new pathogenic pathways that may provide opportunities for early diagnosis and for targets of novel treatments.

C-reactive protein (CRP) is a normal plasma protein that belongs to the pentraxin family, an evolutionary conserved group of proteins involved in acute immunological responses. Levels can rise 100–1000-fold within 24–72 h in a cytokine-mediated response to most forms of tissue injury, infection, or inflammation [6]. In terms of DN, several studies have examined its relationship with inflammation, leading to conflicting results [7–9]. Some data suggests that CRP may be implicated as a risk factor in DN.

TNF-*α* is a pleiotropic cytokine that plays an essential role in mediating inflammatory processes. It is cytotoxic to glomerular, mesangial, and epithelial cells and may induce direct renal damage. Several studies found that diabetic patients with nephropathy have higher serum and urinary concentrations of TNF-*α* than nondiabetic subjects or diabetic patients without renal involvement [10, 11]. 

Local tissue infiltration of monocytes and macrophages is a characteristic of DN. Recent studies have demonstrated that monocyte chemoattractant protein-1 (MCP-1) is a chemotactic cytokine with a high degree of specificity for monocytes and which may be involved in the infiltration of monocytes and macrophages and plays an important role in the progression of DN [12, 13]. Thus, measuring levels of MCP-1 is of important clinical significance in the diagnosis and intervention of early DN.

SAA is an acute phase protein synthesized in the liver and secreted into the blood with a 1000-fold elevation following inflammation. Transforming growth factor-*β* (TGF-*β*) is a cytokine that stimulates the synthesis of acute phase proteins and has been found to be overexpressed in the glomeruli of patients with DN. It is also involved in the induction of extracellular matrix production [14].

As there has been no study done to examine the relationship between inflammatory cytokines and the parameters of UAE, HbA1c, lipids, and blood pressure, the purpose of this study was to detect the levels of hs-CRP, TNF-*α*, and SAA in serum, as well as the levels of uMCP-1 at different stages of DN, while also describing the relationship between these markers and the various parameters.

## 2. Subjects and Methods

### 2.1. Study Subjects

The study was performed on 261 hospitalized patients with T2DM, having an average age of 54.1 years ± 14.2 years. These patients were recruited from the Department of Endocrinology in The First Affiliated Hospital of China Medical University, from September 2011 to November 2012. There were 136 male patients and 125 females. Type 2 diabetes was diagnosed based on the World Health Organization criteria. Patients with cardiac and hepatic diseases, another kidney disease, and infectious diseases were excluded. Patients with a history of diabetic ketoacidosis or hypoglycemic coma during the 3 months preceeding the study were also excluded. None of the patients had an elevated serum creatinine nor used angiotensin-converting enzyme inhibitors (ACEIs) or angiotensin receptor blockers (ARBs). Also, none of the patients used thiazolidinediones or statins. 

Patients were classified into three groups according to urine albumin excretion (UAE) as follows: D1 = normoalbuminuric (patients with urinary albumin levels of <30 mg/g · creatinine (Cr) (112 patients)); D2 = microalbuminuric (patients with microalbuminuria of 30–299 mg/g · Cr (93 patients)); D3 = macroalbuminuria (patients with macroalbuminuria of ≥300 mg/g · Cr (56 patients)). In control group (C), 86 healthy volunteers were also recruited with an average age of 55.2 years ± 12.4 years (45 males, 41 females). The parameters of sex, age, body mass index (BMI), and creatinine were comparable between the study and control groups. General status of the patients and healthy volunteers is shown in Table 1. Informed consents were obtained from the patients before the study began.

### 2.2. Methods

Blood samples were taken before breakfast in the morning (between 8 AM and 11 AM), after an 8 to 12 hour overnight fast. Samples were collected in sterile tubes, centrifuged at 3000 rpm for 15 minutes at 4°C, and then stored at −70°C until assayed. The urine samples were centrifuged at 2000 rpm/min for ten minutes, and a 2 mL supernatant was removed and stored at −70°C. TNF-*α*, SAA, and uMCP-1 were measured by a quantitative sandwich enzyme-linked immunosorbent assay (ELISA). Levels of hs-CRP were measured by immunoturbidimetry. TG, LDL-C, HDL-C, SCr, BUN, and HbA1c were measured in all subjects. Levels of uMCP-1 were expressed as values corrected by the urinary creatinine concentration (milligrams of creatinine/deciliter) to exclude the influence of different urine sample concentrations.

### 2.3. Statistical Analysis

Normally distributed values were analyzed by analysis of variance (ANOVA). Post hoc comparisons of group pairs were performed by Scheffe's multiple comparison test after ANOVA had established significant differences among the groups. Tests of normality between the groups were performed with a Shapiro-Wilk test. Pearson's correlational analysis was used to analyze the levels of inflammation cytokines and various factors. Multiple linear regression analysis and principal component analysis were also used to assess association between lnUAE as a dependent variable and SBP, DBP, lipid,course, HbA1c, uMCP-1, TNF-*α*, hs-CRP, and SAA as independent variables. Analysis of variance and dependability were processed with IBM SPSS, version 12.0. Values were expressed as mean ± SD. *P* values of less than 0.05 were considered statistically significant. 

## 3. Results

### 3.1. Clinical Characteristics of Participants

There were no significant differences between diabetes patients and the control group regarding age, BMI, SCr, BUN, TG, and HDL-C; however, the diabetic patients had higher values of SBP, DBP, TC, LDL-C, and UAE (*P* < 0.05). Among the three diabetes groups there were no significant differences regarding course, SBP, DBP, or TC. However, the levels of HbA1c, LDL-C, and UAE in group D3 were much higher than those in groups D1 and D2 (*P* < 0.05), especially for UAE which was higher in group D2 than in group D1 (*P* < 0.01) (Table 1).

### 3.2. Levels of hs-CRP, TNF-*α*, uMCP-1, and SAA

Levels of hs-CRP, TNF-*α*, uMCP-1, and SAA in groups D1, D2, and D3 were much higher than those in the control group (*P* < 0.05). Among the three diabetes groups, these levels increased consistently with UAE. Levels of hs-CRP, TNF-*α*, uMCP-1, and SAA in group D3 were significantly higher than those in groups D1 and D2 (*P* < 0.01), and the levels in group D2 were elevated compared to those in group D1 (*P* < 0.01) (Table 1).

### 3.3. Correlation Analysis of Inflammation Cytokines and Various Factors

Levels of hs-CRP, TNF-*α*, uMCP-1, and SAA were positively correlated with UAE (*r* = 0.675, *P* < 0.001; *r* = 0.813, *P* < 0.001; *r* = 0.798, *P* < 0.001; *r* = 0.824, *P* < 0.001, resp.), SBP (*r* = 0.431, *P* < 0.001; *r* = 0.522, *P* < 0.001; *r* = 0.427, *P* < 0.001; *r* = 0.615, *P* < 0.001), DBP (*r* = 0.413, *P* < 0.001; *r* = 0.497, *P* < 0.001; *r* = 0.279, *P* < 0.05; *r* = 0.507, *P* < 0.001), LDL-C (*r* = 0.507, *P* < 0.001; *r* = 0.431, *P* < 0.001; *r* = 0.322, *P* < 0.01; *r* = 0.559, *P* < 0.001), and TC (*r* = 0.510, *P* < 0.001; *r* = 0.383, *P* < 0.001; *r* = 0.333, *P* < 0.01; *r* = 0.527, *P* < 0.001), in the T2DM patients. However, there was no significance correlated with course, TG, or HDL-C. It was found that only TNF-*α* was positively correlated with HbA1c (*r* = 0.303, *P* < 0.05) (Table 2).

### 3.4. Regression Analysis and Principal Component Analysis of Inflammation Cytokines and DN

To support the results, linear regression analysis and principal component analysis were performed (Table 3). Using lnUAE as a dependent variable and SBP, DBP, lipids, course, HbA1c, uMCP-1, TNF-*α*, hs-CRP, and SAA as independent variables, it was shown that only constant, HbA1c, principal component for hs-CRP, TNF-*α*, uMCP-1, and SAA had statistical significance (*t* = −4.304, *P* < 0.001; *t* = 2.288, *P* < 0.05; *t* = 13.103, *P* < 0.001, resp.). 

## 4. Discussion

In recent years, several clinical and animal studies have indicated that inflammatory cytokines play an important role in the development and progression of DN [15, 16]. Based on these findings, the present work was designed to investigate the importance of hs-CRP, TNF-*α*, uMCP-1, and SAA in the pathogenesis of DN and thus their use as inflammatory markers for DN development in T2DM.

From our data we found a strong and graded association between CRP and UAE in patients with type 2 diabetes. Plasma concentrations of CRP were significantly higher in subjects with T2DM compared to those without T2DM. Besides other studies [17, 18], the results of our work strongly suggest that inflammation seems to play an important and independent role in early microalbuminuria. Taking into account that inflammation and microalbuminuria are both associated with DN, our results are encouraging for the early recognition and treatment of UAE. 

There are several mechanisms through which CRP may promote DN. First, enhanced renal inflammation may be a mechanism by which CRP promotes diabetic kidney injury. It is well known that nuclear transcription factor-kappa B (NF-*κ*B) is active in many aspects of immune and inflammation responses in human cells. It has been shown that the NF-*κ*B signaling CRP pathway is activated in DN and that CRP is capable of inducing the production of proinflammatory cytokines such as IL-1*β* and TNF-*α* in cultured monocytes or endothelial cells via an NF-*κ*B-dependent mechanism [19–21]. More importantly, CRP itself was induced by high glucose, which, in turn promoted high glucose mediated renal inflammation. This finding suggests that CRP may function as an inflammatory mediator or cofactor of high glucose levels to promote diabetic renal inflammation. This is consistent with previous reports [19, 22].

The present study revealed that serum TNF-*α* levels were significantly increased in diabetic groups when compared with healthy control subjects, which was confirmed by the significant positive correlation between glucose and TNF-*α*. On the other hand, it was observed that there was a significant elevation in serum TNF-*α* values in diabetic microalbuminuric and macroalbuminuric groups in comparison with the diabetic normoalbuminuric group. This was in agreement with the significant positive correlation between TNF-*α* and UAE. 

TNF-*α* is known to stimulate prostaglandin production by mesangial cells and may be responsible for the alteration of glomerular microcirculation. This cytokine also induces endothelial procoagulant activity and increases endothelial permeability [23]. Research in animal models as well as other smaller clinical studies has reported interesting data about the importance of TNF-*α* in the setting of DN [9]. Our results highlighted the possible role of TNF-*α* in the development and progression of renal injury in diabetic patients. We also found that the effect of TNF-*α* on albuminuria did not depend on blood pressure, course, or HbA1c. This suggested that TNF-*α* was an independent factor on DN.

In this study, the level of uMCP-1 was clearly increased in DN. It also appeared earlier than urine microalbumin. It was triggered by increased urinary protein excretion. MCP-1 is a C-C chemokine that exhibits its most potent chemotactic activity toward monocytes. MCP-1 signaling through C-C chemokine receptor type 2 (CCR2) on human mesangial cells has been shown to induce fibronectin mRNA and protein synthesis by a mechanism involving TGF-*β*1 production and activation of NF-*κ*B in these cells, inducing a fibrotic response [24]. 

All of these data suggested that MCP-1 played an important part in the progression and development of DN. In the current study, there was a significant positive correlation between MCP-1 and UAE, which suggested that albuminuria and MCP-1 would be the important risk factors of DN. This was in agreement with the results observed by other authors [25, 26].

SAA is a sensitive acute phase protein which was found to be significantly increased and positively correlated with UAE in Japanese patients with type 2 DN [27]. Dalla Vestra et al. [28] have shown that the levels of SAA and CRP in patients with DN increased in the macroalbuminuric stage and that SAA was positively and significantly correlated with UAE. In this study, we found that levels of SAA in T2DM were elevated compared to those in the controls. They increased consistently with UAE and showed a correlation with UAE in the Pearson correlation analyses. 

As for DN, the most significant risk factors are hyperglycaemia and hypertension. In order to support our results, the linear regression analysis and principal component analysis were performed. We used lnUAE as the dependent variable and blood pressure, lipids, HbA1c, and inflammatory cytokines as the independent variables. We concluded that hs-CRP, TNF-*α*, uMCP-1, and SAA had statistical significance with UAE independent of the conventional risk factors. Our results further confirmed the inflammation theory of DN. Chronic inflammation causes kidney damage in diabetic patients by a variety of ways. Inflammatory factors such as hs-CRP, TNF-*α*, uMCP-1, and SAA constitute a complex cytokine network through which autocrine or paracrine behaviors affect the kidneys due to the expanded effects of these inflammation cascades. 

Studies in DN are fraught with difficulty, given the recognized associations with hypertension and dyslipidemia, both of which are known to influence microcirculation. As expected, in our study an increased prevalence of hypertension occurred in the diabetic groups compared with the control group. Moreover levels of hs-CRP, TNF-*α*, uMCP-1, and SAA were positively correlated with elevated SBP and DBP. This is in agreement with the recent reports made by Morii et al. [25] and may be explained, because hypertension itself is an inflammation reaction. Diabetic patients usually also have lipid disorders. There is research which has shown that TGs and LDL-C are higher and HDL-C is lower in DN groups compared with control groups and non-DN groups. In our study, we found TC and LDL-C were higher in DN groups compared with a control group, especially in the macroalbuminuric group for LDL-C, while TG and HDL-C had no significant difference in these groups. 

We also investigated the correlation between inflammation markers and lipidemia and found that the levels of hs-CRP, TNF-*α*, SAA, and uMCP-1 were positively correlated with TC and LDL-C and had no statistical significance with TG and HDL-C. The reason may be because LDL is easily changed to oxidized low-density lipoprotein (OX-LDL) in DN [29]. Both of them, especially the latter may stimulate the expression of inflammation factors through mesangial cells. We did not find a correlation between inflammation markers and course or HbA1c, but it was present for TNF-*α*. Perhaps the reason was that the patients we selected had no significant difference in course or HbA1c among the three diabetes groups. In conclusion the present study suggested that in type 2 diabetic patients, increased hs-CRP, TNF-*α*, uMCP-1, and SAA were associated with DN pathogenesis. Thus, they may be considered as inflammation markers independent of the conventional risk factors that can be used to estimate the progression of DN. As this was a cross-sectional study, it should be confirmed by further longitudinal research. Also in future, new therapeutic potentials such as anti-CRP, anti-TNF-*α*, anti-MCP-1, or anti-SAA agents could be considered as targets to reduce the risk of renal complications in T2DM.

## Figures and Tables

**Table 1:** Comparison of the general status and study data between diabetes groups and control group.

	C	D1	D2	D3
Number	86	112	93	56
Age (years)	55.2 ± 12.4	54.9 ± 13.1	53.7 ± 12.5	62.6 ± 11.4
BMI (Kg/m^2^)	26.5 ± 3.1	26.3 ± 3.7	26.2 ± 2.9	26.8 ± 3.7
Course (year)		8.9 ± 1.3	9.9 ± 1.7	11.8 ± 2.4
SBP (mmHg)	111.3 ± 10.3	124.0 ± 14.3^b^	130.9 ± 16.9^b^	135.5 ± 17.3^b^
DBP (mmHg)	71.4 ± 8.3	77.8 ± 6.5^b^	82.7 ± 7.8^b^	86.1 ± 14.5^b^
SCr (*μ*mol/L)	63.62 ± 8.79	64.96 ± 15.27	69.02 ± 20.32	78.49 ± 24.12
BUN (mmol/L)	4.09 ± 1.01	6.12 ± 1.31	6.41 ± 1.37	6.76 ± 1.70
HbA1c (%)		7.80 ± 3.28	8.89 ± 2.59	9.97 ± 2.91^c^
TG (mmol/L)	1.69 ± 1.01	1.71 ± 0.97	1.99 ± 1.03	2.13 ± 1.16
TC (mmol/L)	4.33 ± 0.77	5.07 ± 0.83^b^	5.36 ± 1.35^b^	6.40 ± 1.76^b^
LDL-C (mmol/L)	1.92 ± 0.33	3.02 ± 0.67^b^	2.80 ± 1.23^a^	3.97 ± 1.31^bcf^
HDL-C (mmol/L)	1.15 ± 0.12	1.17 ± 0.22	1.13 ± 0.31	1.17 ± 0.30
Hs-CRP (mmol/L)	1.03 ± 0.94	2.41 ± 1.07^a^	3.95 ± 1.18^bd^	4.51 ± 1.89^bdf^
TNF-*α* (mg/mL)	1.01 ± 0.45	1.99 ± 0.56^a^	2.73 ± 0.72^bd^	4.10 ± 0.95^bdf^
UMCP-1/Ucr (ng/mg)	4.51 ± 2.29	24.70 ± 5.37^a^	70.59 ± 18.93^bd^	122.85 ± 63.76^bdf^
SAA (ug/L)	163.90 ± 37.13	318.31 ± 34.35^a^	490.13 ± 37.24^bd^	665.04 ± 64.13^bdf^
Ln (UAE/Ucr)*	2.19 ± 0.60	2.37 ± 0.86^a^	4.08 ± 0.58^bd^	7.34 ± 0.90^bdf^

BMI: body mass index; SBP: systolic blood pressure; DBP: diastolic blood pressure; BUN: blood urea nitrogen; SCr: serum creatinine; HbA1c: glycohemoglobin A1c; TG: triglyceride; LDL-C: low density lipoprotein cholesterol; HDL-C: high density lipoprotein cholesterol; hs-CRP: high sensitivity C-reactive protein; TNF-*α*: tumor necrosis factor alpha; uMCP-1: urinary monocyte chemoattractant protein-1; SAA: serum amyloid-A; UAE/Ucr: urine albumin excretion/urinary creatinine.

^a^ *P* < 0.05, ^b^ *P* < 0.01 diabetic patients versus control; ^c^ *P* < 0.05, ^d^ *P* < 0.01 D2 and D3 versus D1; ^e^ *P* < 0.05, ^f^ *P* < 0.01 D3 versus D2.

*Since the figures of UAE/Ucr were not normally distributed, they were transitioned with ln here (similarly hereinafter).

**Table 2:** Correlation analysis of inflammation cytokines and various factors.

	hs-CRP		TNF-*α*		uMCP-1		SAA	
	*r*	*P*	*r*	*P*	*r*	*P*	*r*	*P*
Age	0.135	0.244	0.194	0.093	0.249*	0.030	0.212	0.065
BMI	0.111	0.340	−0.096	0.409	−0.065	0.575	−0.069	0.555
Course	0.205	0.158	0.141	0.334	0.169	0.247	0.195	0.179
SBP	0.431**	<0.001	0.522**	<0.001	0.427**	<0.001	0.615**	<0.001
DBP	0.413**	<0.001	0.497**	<0.001	0.279*	0.015	0.507**	<0.001
TG	0.178	0.125	0.121	0.296	0.184	0.111	0.112	0.336
HDL-C	−0.120	0.301	−0.154	0.184	−0.175	0.130	−0.120	0.300
LDL-C	0.507**	<0.001	0.431**	<0.001	0.322**	0.005	0.559**	<0.001
TC	0.510**	<0.001	0.383**	<0.001	0.333**	0.003	0.527**	<0.001
HbA1c	0.235	0.104	0.303*	0.034	0.249	0.085	0.198	0.173
Ln (UAE/Ucr)	0.675**	<0.001	0.813**	<0.001	0.798**	<0.001	0.824**	<0.001

**Correlation is significant at the 0.01 level (2-tailed).

*Correlation is significant at the 0.05 level (2-tailed).

**Table 3:** Predictors of proteinuria in DN by multiple linear regression^a,b^.

	Unstandardized coefficients		*t*	*P*
	*B*	Std error		
Constant	−0.357	0.083	−4.304	<0.001
Age	−0.115	0.088	−1.306	0.199
BMI	−0.004	0.081	−0.055	0.956
Course	0.080	0.084	0.948	0.349
HbA1c	0.196	0.085	2.288	0.027
Principal component for SBP and DBP^c^	0.112	0.087	1.298	0.202
Principal component 1 for TG, TC, HDL-C, and LDL-C^d^	0.052	0.077	0.679	0.501
Principal component 2 for TG, TC, HDL-C, and LDL-C^d^	−0.070	0.078	−0.894	0.376
Principal component for hs-CRP, TNF-*α*, uMCP-1, and SAA^e^	1.184	0.009	13.103	<0.001

^a^Dependent variable: ln (UAE/Ucr).

^b^Each variable was standardized by using *Z* scores before being entered into the regression model.

^c^Since the values of SBP and DBP were correlated, their unique principal component was substituted for them in the model and the principal component = 0.928 ∗ SBP + 0.928 ∗ DBP. In the formula, each variable was no longer the original variable, but standardized variable and the coefficients before the standardized variables represented the correlation coefficients of principal component and the corresponding original variables. So this formula showed that SBP and DBP were highly correlated and the extracted component could nearly represent the variables of SBP and DBP.

^d^Since the values of TC, TG, HDL-C, and LDL-C were correlated, their two principal components were substituted for them in the model and the principal component 1 = 0.289 ∗ TG + 0.223 ∗ HDL-C + 0.892 ∗ LDL-C + 0.919 ∗ TC, the principal component 2 = 0.770 ∗ TG − 0.793 ∗ HDL-C − 0.090 ∗ LDL-C + 0.128 ∗ TC. In the formulas, each variable was no longer the original variable but standardized variable and the coefficients before the standardized variables represented the correlation coefficients of principal component and the corresponding original variables. So formula 1 showed that LDL-C and TC were highly correlated and component 1 could represent the variables of LDL-C and TC, while formula 2 showed that TG and HDL-C were highly correlated and component 2 could represent the variables of TG and HDL-C.

^e^Since the values of hs-CRP, TNF-*α*, uMCP-1, and SAA were correlated, their unique principal component was substituted for them in the model and the principal component = 0.841 ∗ hs-CRP + 0.928 ∗ TNF-*α* + 0.883 ∗ uMCP-1 + 0.944 ∗ SAA. In the formula, each variable was no longer the original variable, but standardized variable and the coefficients before the standardized variables represented the correlation coefficients of principal component and the corresponding original variables. Since only one principal component was extracted among the four inflammatory factors and the correlation coefficients were all close to 1, it showed that the four inflammatory factors were highly correlated and the component could almost contain all the information of the four variables.
